The article "Machine Learning-Based Psychology Evaluation of College Students for Building Innovative Health Service System" was published in 2022. Journal: J Environ Public Health.

# Machine Learning-Based Psychology Evaluation of College Students for Building Innovative Health Service System

**DOI:** 10.1155/2022/6302756

**Published:** 2022-09-27

**Authors:** Xi Zhang

**Affiliations:** Academic Affaires Office, Shangqiu Polytecnic, ShangQiu 476001, China

## Abstract

Leadership psychology among college students is a multidimensional concept that primarily encompasses practical ability, teamwork ability, political literacy, emotional intelligence, etc. At present, a common problem among the surveyed college students is their leadership ability is not strong. Reasons include the lack of leadership-related knowledge and leadership awareness among college students as well as the fact that the public, particularly college educators, do not give leadership training a sufficient attention. Leadership psychology is a primary factor influencing the development of college students. It is necessary to strengthen college students' leadership education. This work extracts the key factors that influence the leadership of college students by analyzing their big behavior data. The extracted factors include the theoretical knowledge of leadership, practical ability, leadership psychology, home education, and exercise. To evaluate the degrees of these factors influencing the students' leadership, we develop an advanced multicriteria decision-making framework based on the ENtropy theory and the Technique for Order of Preference by Similarity to Ideal Solution (TOPSIS), called EN-TOPSIS. In EN-TOPSIS, an entropy method is used to determine the criteria weights rather than using the subjective weighting method. Three groups of college students are surveyed and evaluated based on the five factors. Each group contains ten students. The evaluation results show that the leadership of the students is mainly influenced by their practical ability and leadership psychology. The students with the highest evaluation score are recognized as having high levels of leadership.

## 1. Introduction

College students' leadership is a multidimensional concept, which mainly includes practical ability, teamwork ability, political literacy, emotional intelligence, self-management, and leadership psychology [1]. At present, a common problem among the surveyed college students is their leadership psychology is not strong. Reasons include the lack of leadership-related knowledge and leadership psychology of college students. And the fact that the public, especially college educators, do not pay enough attention to leadership psychology training. Leadership psychology is a primary factor influencing the development of college students. It is necessary to strengthen college students' leadership education. In the past few years, more and more attention has been paid to the leadership problems on college students [2]. The leadership problems of students have been reported all over the world, and the leadership of college students is not in a well condition. College leadership is a serious problem and will affect their study experience in college. Leadership problems can even affect students' legal behaviors and their future life.

In this paper, we will investigate using multicriteria decision-making (MCDM) technologies to evaluate which leadership elements can affect students' leadership with legal constraints. MCDM refers to the decision making in the set of conflicting and noncommensurable schemes [3]. Multiple criteria should be considered when making decisions, which is one of the important contents in the field of decision analysis. Noncommensurable between objectives and inconsistency of measurement categories, that is, there is no unified measurement standard or unit of measurement for each objective, so it is difficult to compare. According to whether the decision-making scheme is finite or infinite, MCDM is divided into multiple objectives and multiple attribute decision making [4]. Multiobjective decision-making is a MCDM problem that has nondiscrete decision variables and unconstrained decision schemes [5].

TOPSIS is a ranking method based on the proximity between the idealized target and the evaluation objects [6]. It is a distance-based evaluation method. Its primary idea is to calculate the distance between the positive and negative ideal solutions and the evaluating samples and calculate the relative closeness to the ideal solutions. If a sample is close to the negative ideal solution, then it is farther away from the positive ideal solution. The pros and cons of each alternative can be evaluated. TOPSIS is one of the most effective ranking methods for MCDM with limited alternatives and criteria. TOPSIS reduces the influence of different criterion dimensions after deal with the original normalized data. It can use the information of the source data. Therefore, it can completely indicate the gap between alternatives by considering the actual situation. It has the advantages of reliability, intuition, and authenticity. In addition, it does not have specific requirements for sample data.

Compared with the single index mutual analysis method, TOPSIS method can centrally reflect, analyze, and evaluate the overall situation. It has universal applicability. For example, it can be used to evaluate health quality, planned immunization work quality, and medical quality [7]. It can evaluate the setting of professional courses, customer satisfaction, software project risk assessment, and real estate investment site selection. It has been widely and systematically used to evaluate the economic benefits of enterprises, the macroeconomic benefits between cities, the competitiveness of regional science and technology [8], and the well-off society in rural areas. However, there are still various problems of TOPSIS for decision making. For example, the weight information should be given in advance, so the result is subjective. In addition, this method has the reverse order problems due to the occurrence of the new criteria or alternatives in application, which needs to be analyzed and studied more specifically and deeply [9].

This work extracts the key factors that influence the leadership of college students by analyzing the big behavior data of college students. The extracted factors include the theoretical knowledge of leadership, practical ability, leadership psychology, home education, and exercise. To evaluate the degrees of these factors influencing the students' leadership, we develop an advanced MCDM framework based on the Technique for Order of Preference by Similarity to Ideal Solution (TOPSIS), called EN-TOPSIS. In EN-TOPSIS. The principal contributions of EN-TOPSIS are as follows:

1. *Use an Entropy Method to Determine the Criteria Weights Rather than Using the Subjective Weighting Method*. Therefore, EN-TOPSIS can analyze and research problems more objectively
2. *Survey and Evaluate Three Groups of College Students Based on the Five Factors*. Each group contains ten students. The evaluation results show that the leadership of the students is mainly influenced by their practical ability and leadership psychology. The students with the highest evaluation score are recognized as having high levels of leadership

The remaining paper is arranged as follows: Section 2 introduces the related work about the MCDM technologies and their application in leadership evaluation.  Section 3 presents the technical details of EN-TOPSIS.  Section 4 shows an experiment to use the proposed EN-TOPSIS to evaluate leadership of college students.  Section 5 concludes this work and describes future research directions.

## 2. Related Work

Vafaei et al. [10] proposed that in MCDM, standardization must change criteria values into a universal scale to rate and rank alternatives. The authors' research contribution is to assess the assessment methods for standardization techniques and the proposed assessment process is the best normalization technique used in TOPSIS to obtain a more robust assessment and selection. A work by Muhsen et al. [11] uses load management to save energy and focuses on a multiobjective optimized differential evolution (MODE) algorithm to obtain an optimal set of user load management by simultaneously minimizing energy costs and user inconvenience. The optimal set of solutions obtained is ranked from the most outstanding to the worst using the MCDM method, which uses a mixture of the Analytic Hierarchy Process (AHP) with the TOPSIS to ensure that energy costs and peak consumption are saved while maintaining an adequate range of customer nuisance. In the work of Dutta et al. [12], an algorithm is designed to find a set of criteria by which the rank of another alternative can be obtained by changing the criteria of one alternative. The behavior of the closeness coefficients of the alternates when the criterion scores are changed is investigated and two algorithms are provided to identify high and low order realizable alternatives. Subsequently, the rank inversion of a couple of alternates is described and the concept of rank-sensitive intervals is introduced. Finally, the validity of the model is verified using university rankings as an example. The purpose of the work of Akram et al. [13] is to extend the TOPSIS method to a multiobjective clustering resolution problem based on Pythagorean fuzzy data. A Pythagorean fuzzy decision matrix is used for information evaluation. The alternatives are ranked using a modified closeness index to determine the optimal alternative.

In the work of Chauhan et al. [14], the fuzzy TOPSIS method was used to pick out the risks connecting the agricultural sector in India based on a review of the literature, and an analysis of the constitution makers' works on mental work stress and pressure where all identified risk factors are ranked according to actual local preferences. QFD techniques were then applied to propose design parameters to minimize farmers' work stress. The work of Liu et al. [15] evaluates the emergency response capability of university students based on the TOPSIS creative algorithm questionnaire. First, the survey method was used to evaluate the current cases of university students' response capability towards emergencies. The TOPSIS-based evaluation algorithm was developed to assess the crisis response capability of university students. The reasons for the shortage of students' emergency response capability were studied based by the reviews results. At the same time, the development countermeasures for the cultivation of college students' crisis response skill are proposed. A study by Omid et al. [16] investigated the impact of security climate and psychosocial safety climate elements on the safety performance of employees in the process industry. The collected data perform average analysis of the MCDM approach. Scenarios were also ranked using the TOPSIS. The results indicate that safety professionals need to consider the climate factors of psychosocial safety to improve the performance in facilities in high hazard processes. The work of Han et al. [17] proposes a vague approach to the clinical diagnosis of yin and yang bipolar disorder based on a group decision-making process incorporating multiple criteria. It introduces a group decision-making process based on multiple criteria for the diagnosis of bipolar disorder. The complexity of bipolar disorder is described by examining the interrelationships between symptoms.

The paper by Dandage et al. [18] uses the TOPSIS method to collect TOPSIS data to rank the main danger types in international projects. The results show that the TOPSIS method ranks political risk, technical risk, and design-related risk as the first three risk types in international projects. This work offers an overview of the risk types in international projects, and the results of their ranking show that it can help in developing strategies to deal with the risks appropriately. In the paper of Mo et al. [19], a risk assessment system is proposed. The system is designed to model many trial risks based on qualitative information in judicial databases. An extension technique has been introduced into the system to accommodate this complexity. The work of Radovanović et al. [20] performed an adaptation of the commonly used decision-making method which is the TOPSIS method to generate utility scores in the absence of differential impact. The results show the validity of the solution solutions shown on the synthetic dataset, as well as on the sample dataset on criminal justice.

EN-TOPSIS is an advanced MCDM framework based on TOPSIS, which can analyze and research problems more objectively. What makes EN-TOPSIS special compared to common evaluation methods is that EN-TOPSIS uses an entropy method to determine standard weights instead of subjective weighting methods. Therefore, EN-TOPSIS can make more reasonable decisions and can effectively solve the problem of reverse order.

## 3. EN-TOPSIS: An Efficient TOPSIS for Evaluating Legal Consciousness Based on Leadership Psychology of Students

Multiattribute decision analysis is used to establish an evaluation index system, determine a set of alternatives, and collect data based on the principles of problem completeness, scientificity, data availability, and operability. The objective data is then processed through the selected method. By integrating schemas, the intuitive reflection of each alternative is obtained. It can help decision makers to make accurate decisions.

For a problem, decision makers need to comprehensively consider from multiple aspects. They should summarize and merge all aspects to form a set of criteria, denoted as *C* = {*c*^1^, *c*^2^, ⋯*c*^*m*^}, where *m* is the criterion number. The set of decision options or alternatives is denoted as *A* = {*a*^1^, *a*^2^, ⋯*a*^*n*^}, where *n* is the alternative number. Therefore, a decision matrix of *m* × *n* is composed of the criteria and the alternatives.

After the decision matrix is constructed, the natural attribute value needs to be processed, and the natural attribute value *t*_*j*_^*i*^ is changed to the corresponding preference representation value *v*_*j*_^*i*^, denoted as *v*(*a*^*i*^) = (*v*_1_^*i*^, ⋯*v*_*m*_^*i*^). The most common transformations include the transformation of fuzzy language into numbers and the standardization of numerical values in different dimensions.

Weights are then assigned to all criteria. The more important criteria have greater weights, the weight vector of the criterion set can be recorded as *w* = (*w*_1_, ⋯*w*_*j*_, ⋯*w*_*m*_) and requires ∑_*j*=1_^*m*^*w*_*j*_ = 1. Finally, a mapping function G is constructed, and the weight and preference representation vectors are integrated into the evaluation result value of the alternative *a*^*i*^. Generally, the most used mapping function G is the weighting function.

The TOPSIS method, called EN-TOPSIS, is a sorting algorithm that approximates the ideal solution. It calculates the distance between the current evaluation object with the ideal and anti-ideal points, respectively. The closer to the positive point and the farther from the negative point, the better the performance. The calculation steps of TOPSIS are as follows:

1. *Data Normalization*. Since the dimensions of different criteria may be different, to eliminate the influence of different dimensions on the results, it is necessary to standardize the data first. The standardization generally includes vector normalization, sum normalization, and maximum and minimum normalization, where vector normalization is performed

(1) $$\begin{array}{c} v_{j}^{i}=\frac{t_{j}^{i}}{\sqrt{\sum_{i=1}^{n}{\left(t_{j}^{i}\right)}^{2}}}, \end{array}$$

where  *t*_*j*_^*i*^ is the natural attribute value of the alternative *i* under the criterion *j*, and *n* is the alternative number.

(2) *Find the Ideal Pointa*^+^*and the Anti-Ideal Pointa*^−^. For the benefit criteria, the ideal point *a*^+^ is the maximum value among all alternatives with respect to criterion *j*, and the anti-ideal point *a*^−^ is the minimum value among all alternatives under criterion *j*, denoted by

(2) $$\begin{array}{c} v_{j}\left(a^{+}\right)=\max_{i=1}^{n}v_{j}^{i}, \end{array}$$

(3) $$\begin{array}{c} v_{j}\left(a^{-}\right)=\min_{i=1}^{n}v_{j}^{i}. \end{array}$$

As for the cost criteria, the values of the anti-ideal and ideal points are just opposite to the benefit criteria.

(3) *Calculate the Distance Between the Anti-Ideal and the Ideal Points of the Alternativea*^*i*^*Under the Indexj*. When calculating the distance, we used a normalization factor *θ*_*j*_^+^ and the anti-ideal point normalization factor *θ*_*j*_^−^, then the distances are calculated by

(4) $$\begin{array}{c} d_{j}^{+}\left(a^{i}\right)=\frac{\left|t_{j}\left(a^{+}\right)-t_{j}\left(a^{i}\right)\right|}{\theta_{j}^{+}}, \end{array}$$

(5) $$\begin{array}{c} d_{j}^{-}\left(a^{i}\right)=\frac{\left|t_{j}\left(a^{-}\right)-t_{j}\left(a^{i}\right)\right|}{\theta_{j}^{-}}, \end{array}$$

where *θ*_*j*_^+^ = max{max{|*t*_*j*_(*a*^+^) − *t*_*j*_(*a*^*i*^)|: *i* = 1, 2, ⋯, *n*}, |*t*_*j*_(*a*^+^) − *t*(*a*^−^)|} and *θ*_*j*_^−^ = max{max{|*t*_*j*_(*a*^−^) − *t*_*j*_(*a*^*i*^)|: *i* = 1, 2, ⋯, *n*}, |*t*_*j*_(*a*^+^) − *t*_*j*_(*a*^−^)|}.

The monotonic and nonmonotonic criteria are uniformly processed. The monotonic criterion is a criterion for evaluating both single winner and multiple winners scored election systems. A scored system of voting is monotonic when neither preventing the election of an applicant by ranking them higher on some voter rolls nor electing an unaccountable applicant by scoring them lower on some voter rolls is feasible. This is a form of preference expression for each indicator. Through such processing, the objective value becomes the preference value of the decision maker.

(4) *Determine Weights for Criteria*. When the mutual importance between the criteria is not clear, the entropy method can be used for weighting. Since the entropy method is very mature, this article will not go into details. When the mutual importance of the criteria weights is clear, but the specific weights are unknown, the following two methods can be used.

At first, the weights of criteria are calculated based on the data envelopment method. Based on the observation data, the decision-making unit is evaluated by the change weight, so that the weight of the index is changed when this method is used. That is, under different alternatives, the weights are different, and the optimization model is shown as

(6) $$\begin{array}{c} \mathrm{Max}\frac{D{\left(a^{i}\right)}^{-}}{D{\left(a^{i}\right)}^{-}+D{\left(a^{i}\right)}^{+}}. \end{array}$$

If the rank of alternative *i* under qualitative criterion *j* is *s*_*u*_, the optimization model is calculated by

(7) $$\begin{array}{c} \frac{u-1}{t}\leq d_{j}^{0}{\left(a^{i}\right)}^{+}\leq \frac{s}{t}, \end{array}$$

(8) $$\begin{array}{c} \frac{t-u+1}{t}\leq d_{j}^{0}{\left(a^{i}\right)}^{-}\leq \frac{t-u}{t}, \end{array}$$

(9) $$\begin{array}{c} w_{i}-w_{j}=t, \end{array}$$

(10) $$\begin{array}{c} \overset{q}{\underset{j=1}{\sum }}w_{j}=1, \end{array}$$

where *t* is a constant, indicating how much the criterion *i* is more important than the criterion *j*. This optimization model is solved for each alternative to get different weights.

(5) *Fix Weights for All Alternatives*. It is practical to change the weights under different alternatives, but it increases the amount of calculation. To uniformly weight the criteria, the optimization model is shown as

(11) $$\begin{array}{c} \mathrm{Max}\overset{n}{\underset{i=1}{\sum }}\frac{D{\left(a^{i}\right)}^{-}}{D{\left(a^{i}\right)}^{-}+D{\left(a^{i}\right)}^{+}}, \end{array}$$

(12) $$\begin{array}{c} \forall a^{i}\in A,\frac{u-1}{t}\leq d_{j}^{0}{\left(a^{i}\right)}^{+}\leq \frac{u}{t}, \end{array}$$

(13) $$\begin{array}{c} \frac{u-t+1}{u}\leq d_{j}^{0}{\left(a^{i}\right)}^{-}\leq \frac{u-t}{t}. \end{array}$$

(6) *Calculate the Distance Between Each Alternative with the Ideal and the Anti-Ideal Points, Respectively*.

(14) $$\begin{array}{c} D{\left(a^{i}\right)}^{+}={\left\{\overset{m}{\underset{j=1}{\sum }}w_{j}d_{j}^{+}{\left(a^{i}\right)}^{h}\right\}}^{1/h}, \end{array}$$

(15) $$\begin{array}{c} D{\left(a^{i}\right)}^{-}={\left\{\overset{m}{\underset{j=1}{\sum }}w_{j}d_{j}^{-}{\left(a^{i}\right)}^{h}\right\}}^{1/h}. \end{array}$$

(7) *Calculate the Closeness of Alternatives to the Ideal Point*

(16) $$\begin{array}{c} D\left(a^{i}\right)=\frac{D{\left(a^{i}\right)}^{-}}{D{\left(a^{i}\right)}^{-}+D{\left(a^{i}\right)}^{+}}. \end{array}$$

The larger the value of *D*(*a*^*i*^), the better the solution.

## 4. Experiment

### 4.1. Evaluation Settings

We use an example to describe the process of using TOPSIS for decision making. Three groups of students are surveyed. Each group contains ten students. They are evaluated in terms of five criteria: the theoretical knowledge of leadership (c1), practical ability (c2), leadership psychology (c3), home education (c4), and exercise (c5). Each criterion is ranked by using the scores in references [1, 8].  Table 1 shows the different scores of each member of the 3 groups of students under the 5 criteria. a1 to a10 represent 10 students.

### 4.2. Analysis of Results

The research team believes that the relative importance among the 5 criteria is clear.  Table 2 shows that the ideal points of c1~c5 of Group 1 are 9, 10, 8, 10, and 10, respectively. The anti-ideal points are 4, 3, 2, 2, and 2, respectively. The ideal point consists of all possible best criteria values, while the anti-ideal point consists of all possible worst criteria values. The ideal points of c1~c5 of Group 2 are 8, 10, 10, 10, and 8, respectively. The anti-ideal points are 2, 2, 2, 2, and 2, respectively. For Group 3, the ideal points for criteria c1~c5 are 10, 8, 8, 8, and 10, respectively. The anti-ideal points are 4, 2, 4, 2, and 2, respectively.

Based on the proposed TOPSIS algorithm, the evaluation scores and ranking results are shown in Tables 3–5 for Group 1, Group 2 and Group 3, respectively. In Tables 3–5, marks represent the evaluation scores, and ranks represent the ranking of the evaluation scores from high to low.

From Tables 3–5, we can see that the ranking results are similar regardless of the value of *h*. In Group 1, student a9 has the most serious problem based on the mental factors of their theoretical knowledge of leadership, practical ability, leadership psychology, home education, and exercise. In Group 2, student a1 has the most serious problem among all the 10 students. In Group 3, student a3 has serious leadership problem in terms of the five leadership investigating factors. Overall, the practical ability and leadership psychology of the students are mainly influenced by their leadership.

## 5. Conclusion

In this work, we first determined the key factors that influence the leadership psychology of college students by analyzing the big behavior data of college students. The extracted factors include the theoretical knowledge of leadership, practical ability, leadership psychology, home education, and exercise. To evaluate the degrees of these factors influencing the students' leadership, we developed an advanced MCDM framework called EN-TOPSIS. In EN-TOPSIS, an entropy method was used to determine the criteria weights rather than using the subjective weighting method. Three groups of college students were surveyed and evaluated based on the five factors. Each group contained ten students. The experiment evaluation performance shows that the leadership of the students is mainly influenced by their practical ability and leadership psychology. The students with the highest evaluation score were recognized as having high levels of leadership. However, EN-TOPSIS requires a lot of preprocessing work, and the weight update process is complicated. In the future, more deep learning-based methods can be introduced to evaluate scores. Evaluation methods based on deep learning can make evaluation more intelligent and accurate.

## Figures and Tables

**Table 1:** Decision matrix.

Alternatives		a1	a2	a3	a4	a5	a6	a7	a8	a9	a10
Group 1	c1	8	4	5	4	6	8	6	7	6	9
	c2	4	4	10	6	4	6	9	6	8	3
	c3	6	8	6	4	2	6	4	6	8	4
	c4	8	8	10	2	4	6	2	4	4	8
	c5	2	10	8	4	6	6	4	2	2	2

Group 2	c1	8	8	6	4	6	8	6	6	2	2
	c2	6	2	10	6	2	6	8	8	4	10
	c3	10	8	6	4	2	8	6	6	8	8
	c4	8	2	8	2	4	6	4	6	10	4
	c5	6	4	8	2	6	8	2	2	2	4

Group 3	c1	6	10	6	4	8	10	6	6	8	6
	c2	4	2	8	6	2	6	8	6	6	8
	c3	8	6	6	4	4	8	4	4	4	6
	c4	6	4	8	2	2	6	2	6	4	4
	c5	4	4	10	7	5	8	7	6	2	5

**Table 2:** The setting of ideal point and anti-ideal point.

	c1	c2	c3	c4	c5
Group 1					
Ideal point	9	10	8	10	10
Anti-ideal point	4	3	2	2	2
Group 2					
Ideal point	8	10	10	10	8
Anti-ideal point	2	2	2	2	2
Group 3					
Ideal point	10	8	8	8	10
Anti-ideal point	4	2	4	2	2

**Table 3:** Evaluation scores and ranking results for Group 1.

	*h* = 0.1		*h* = 0.8		*h* = 1		*h* = 2	
	Marks	Ranks	Marks	Ranks	Marks	Ranks	Marks	Ranks
a1	0.7824	3	0.7768	2	0.7195	4	0.7376	4
a2	0.4722	8	0.4394	6	0.4843	6	0.4415	8
a3	0.7519	4	0.7605	3	0.6157	5	0.7224	5
a4	0.4236	9	0.3242	9	0.3250	9	0.3503	9
a5	0.3478	10	0.2898	10	0.2867	10	0.3490	10
a6	0.7501	5	0.7172	5	0.7831	2	0.7388	3
a7	0.5382	7	0.4288	7	0.4775	7	0.4925	7
a8	0.5727	6	0.4039	8	0.4382	8	0.5620	6
a9	0.8001	2	0.7321	4	0.7459	3	0.7450	2
a10	0.8235	1	0. 8647	1	0.8928	1	0.8399	1

**Table 4:** Evaluation scores and ranking results for Group 2.

	*h* = 0.1		*h* = 0.8		*h* = 1		*h* = 2	
	Marks	Ranks	Marks	Ranks	Marks	Ranks	Marks	Ranks
a1	0. 8593	1	0.8283	1	0.8688	1	0.8027	1
a2	0.4673	7	0.4653	7	0.4743	6	0.4295	6
a3	0.6765	5	0.6786	5	0.6367	5	0.6729	5
a4	0.3216	9	0.3126	9	0.3208	9	0.3433	9
a5	0.2254	10	0.2218	10	0.2724	10	0.2372	10
a6	0.7128	4	0.7819	2	0.7792	2	0.7321	2
a7	0.4189	8	0.4272	8	0.4549	8	0.4017	8
a8	0.4786	6	0.5148	6	0.4687	7	0.4185	7
a9	0.7864	2	0.7054	3	0.7195	4	0.7155	3
a10	0.7605	3	0.7001	4	0.7238	3	0.7010	4

**Table 5:** Evaluation scores and ranking results for Group 3.

	*h* = 0.1		*h* = 0.8		*h* = 1		*h* = 2	
	Marks	Ranks	Marks	Ranks	Marks	Ranks	Marks	Ranks
a1	0.7864	2	0.7054	3	0.7195	4	0.7155	3
a2	0.4673	7	0.4653	7	0.4743	6	0.4295	6
a3	0. 8593	1	0.8283	1	0.8688	1	0.8027	1
a4	0.3216	9	0.3126	9	0.3208	9	0.3433	9
a5	0.2254	10	0.2218	10	0.2724	10	0.2372	10
a6	0.7128	4	0.7819	2	0.7792	2	0.7321	2
a7	0.4189	8	0.4272	8	0.4549	8	0.4017	8
a8	0.4786	6	0.5148	6	0.4687	7	0.4185	7
a9	0.6765	5	0.6783	5	0.6367	5	0.6729	5
a10	0.7605	3	0.7001	4	0.7238	3	0.7010	4

## Data Availability

The experimental data used to support the findings of this study are available from the corresponding author upon request.

## References

[1] Gianfredi V., Balzarini F., Gola M. (2019). Leadership in public health: opportunities for young generations within scientific associations and the experience of the “Academy of young leaders”. *Frontiers in Public Health*.

[2] Pedrelli P., Nyer M., Yeung A., Zulauf C., Wilens T. (2015). College students: mental health problems and treatment considerations. *Academic Psychiatry: the Journal of the American Association of Directors of Psychiatric Residency Training and the Association for Academic Psychiatry*.

[3] Sun L., Zhou R., Peng D., Bouguettaya A., Zhang Y. (2022). Automatically building service-based systems with function relaxation. *IEEE Transactions on Cybernetics*.

[4] Reshetnikov V. A., Tvorogova N. D., Hersonskiy I. I., Sokolov N. A., Petrunin A. D., Drobyshev D. A. (2020). Leadership and emotional intelligence: current trends in public health professionals training. *Frontiers in Public Health*.

[5] Huang S., Liu A., Zhang S., Wang T., Xiong N. N. (2021). BD-VTE: a novel baseline data based verifiable trust evaluation scheme for smart network systems. *IEEE Transactions on Network Science and Engineering*.

[6] Dhanani L. Y., Franz B. (2020). The role of news consumption and trust in public health leadership in shaping COVID-19 knowledge and prejudice. *Frontiers in Psychology*.

[7] Horváth C., Hong K., Wheeler P. (2022). How management and leadership training can impact a health system: evaluation findings from a public health management training program in Cambodia. *Frontiers in Public Health*.

[8] Xu X., Arshad M. A., Mahmood A. (2021). Talent competitiveness evaluation of the Chongqing intelligent industry based on using the entropy TOPSIS method. *Information*.

[9] Liern V., Pérez-Gladish B. (2022). Multiple criteria ranking method based on functional proximity index: un-weighted TOPSIS. *Annals of Operations Research*.

[10] Vafaei N., Ribeiro R. A., Camarinha-Matos L. M. (2018). Data normalisation techniques in decision making: case study with TOPSIS method. *International Journal of Information and Decision Sciences*.

[11] Muhsen D. H., Haider H. T., Al-Nidawi Y. M., Khatib T. (2019). Domestic load management based on integration of MODE and AHP-TOPSIS decision making methods. *Sustainable Cities and Society*.

[12] Dutta B., Singha T., Goh M., Lamata M. T., Verdegay J. L. (2019). Post factum analysis in TOPSIS based decision making method. *Expert Systems with Applications*.

[13] Akram M., Dudek W. A., Ilyas F. (2019). Group decision-making based on pythagorean fuzzy TOPSIS method. *International Journal of Intelligent Systems*.

[14] Chauhan H., Satapathy S., Sahoo A. K. (2021). A QFD approach based on fuzzy TOPSIS to reduce the mental stress of farmers. *International Journal of Service Science, Management, Engineering, and Technology (IJSSMET)*.

[15] Liu Y., Zhou W., Song Y. (2021). Evaluation of college students’ emergency response capability based on questionnaire-TOPSIS innovative algorithm. *Complexity*.

[16] Omidi L., Salehi V., Zakerian S. A., Nasl Saraji J. (2022). Assessing the influence of safety climate-related factors on safety performance using an integrated entropy-TOPSIS approach. *Journal of Industrial and Production Engineering*.

[17] Han Y., Lu Z., Du Z., Luo Q., Chen S. (2018). A YinYang bipolar fuzzy cognitive TOPSIS method to bipolar disorder diagnosis. *Computer Methods and Programs in Biomedicine*.

[18] Dandage R., Mantha S. S., Rane S. B. (2018). Ranking the risk categories in international projects using the TOPSIS method. *International journal of managing projects in business*.

[19] Mo H., Yong Q., Liu N. Trial risk index model and assessment system based on extended TOPSIS method.

[20] Radovanović S., Petrović A., Delibašić B., Suknović M. Eliminating Disparate Impact in MCDM: The case of TOPSIS.

